# Pharmacokinetics and *in vitro* efficacy of salicylic acid after oral administration of acetylsalicylic acid in horses

**DOI:** 10.1186/s12917-017-0955-1

**Published:** 2017-01-19

**Authors:** Kathrin Buntenkötter, Maren Osmers, Ina Schenk, Wilhelm Schänzer, Marc Machnik, Michael Düe, Manfred Kietzmann

**Affiliations:** 1 Institute of Pharmacology, Toxicology and Pharmacy, University of Veterinary Medicine Hannover Foundation, Hannover, Germany; 2 Institute for Biochemistry, German Sport University, Cologne, Germany; 3 Sassenberg, Germany

**Keywords:** Acetylsalicylic acid, Salicylic acid, COX-inhibition, Pharmacokinetics, Horses

## Abstract

**Background:**

Although acetylsalicylic acid (ASA) is not frequently used as a therapeutic agent in horses, its metabolite SA is of special interest in equestrianism since it is a natural component of many plants used as horse feed. This led to the establishment of thresholds by horse sport organizations for SA in urine and plasma. The aim of this study was to investigate plasma and urine concentrations of salicylic acid (SA) after oral administration of three different single dosages (12.5 mg/kg, 25 mg/kg and 50 mg/kg) of acetylsalicylic acid (ASA) to eight horses in a cross-over designed study.

**Results:**

In the 12.5 mg/kg group, SA concentrations in urine peaked 2 h after oral administration (2675 μg/mL); plasma concentrations peaked at 1.5 h (17 μg/mL). In the 25 mg/kg group, maximum concentrations were detected after 2 h (urine, 2785 μg/mL) and 1.5 h (plasma, 23 μg/mL). In the 50 mg/kg group, maximum concentrations were observed after 5 h (urine, 3915 μg/mL) and 1.5 h (plasma, 45 μg/mL). The plasma half-life calculated for SA varied between 5.0 and 5.7 h. The urine concentration of SA fell below the threshold of 750 μg/mL (set by the International Equestrian Federation FEI and most of the horseracing authorities) between 7 and 26 h after administration of 12.5 and 25 mg/kg ASA and between 24 and 36 h after administration of 50 mg/kg ASA. For ASA, IC_50_ were 0.50 μg/mL (COX-1) and 5.14 μg/mL (COX-2). For salicylic acid, it was not possible to calculate an IC_50_ for either COX due to insufficient inhibition of both cyclooxygenases.

**Conclusion:**

The established SA thresholds of 750 μg//mL urine and 6.5 μg/mL plasma appear too generous and are leaving space for misuse of the anti-inflammatory and analgetic compound ASA in horses.

## Background

Salicylic acid (SA) is one of the oldest nonsteroidal anti-inflammatory drugs (NSAIDs) and has been used as an antipyretic agent and in acute rheumatic events in humans for a long time [1]. Also in veterinary medicine, it has been administered in cases of joint disease in dogs and horses [2]. Acetylsalicylic acid (ASA) was synthesized to have the same effects as SA with an improved gastric and systemic tolerability profile [3]. After administration, ASA is rapidly converted to SA [4]. Additionally, ASA is sensitive to methanol, heat, change of pH and other factors. So, ASA itself cannot be detected with sufficient accuracy, because it is dissociated to SA and acetylic acid, even during sample storage and LC-MS analysis. Even though ASA is not frequently used as a therapeutic agent in horses, its metabolite SA is of special interest in equestrianism since it is a natural component of many plants used as horse feed, e.g. alfalfa hay or willow bark. Therefore, SA concentrations can be found in blood and urine samples of horses after consumption of any of these plants [5]. This led to the establishment of thresholds by horse sport organizations for SA in urine and plasma to avoid positive doping cases due to accidental feed intake, resulting in false positive. The International Equestrian Federation (FEI) and most of the horseracing authorities (for example in Europe, U.S.A.) have set SA thresholds at 750 μg/mL in urine and 6.5 μg/mL in plasma [6]. These threshold levels were based on several studies [5, 7, 8], in which the average urine concentration of SA was dependent on the horse’s diet and country of origin. However, the thresholds were established on a arbitrary statistical basis and not extrapolated from any irrelevant plasma or urine concentration as proposed by Toutain and Lassourd [9].

The study presented aimed to investigate average time intervals elapsed until plasma and urine concentrations fall below the threshold after oral administration of different dosages of ASA. Recommended ASA dosages for horses in literature vary between 5 and 100 mg/kg and from twice daily to every other day [10]. Main indications are inflammatory processes, pain and fever. In this cross-over designed study, eight horses received 12.5 mg/kg, 25 mg/kg, and 50 mg/kg ASA orally once daily. Blood and urine samples were analyzed via HPLC-MS/MS. Furthermore, to assess the efficacy of salicylates on COX-1 and COX-2 inhibition in horses, the IC_50_, i.e. the drug concentration required to inhibit 50% of COX activity *in vitro*, was determined for ASA and SA in a whole blood assay.

## Methods

### Pharmacokinetic study

#### Animals

The animal study protocol was approved by the regional administration of the governmental body (LAVES; Lower Saxony, Germany; 33.9-42502-04-11/0512). Eight standardbred horses (4 mares, 4 geldings, 12.4 ± 3.2 years old; 656 ± 95 kg body weight) were used in this study. Horses were housed in stables of Serumwerk Memsen, WDT, Germany (owner of the horses) with straw bedding and daily turnout. They were fed a diet free from detectable SA contamination consisting of hay, grass, beets and water *ad libitum*. All horses were healthy on the basis of a clinical examination prior to the study.

#### Animal study

Three dosages of ASA were chosen: 12.5 mg/kg, 25 mg/kg, and 50 mg/kg bodyweight once daily. Horses received single oral doses of the ASA powder (Pyrinagil®, Veyx, Schwarzenborn, Germany) mixed with syrup in 100 mL syringes. The study was conducted in a 4-way, 3-treatment cross-over design with a washout period of at least 2 weeks. Blood samples were drawn in lithium heparin tubes at the following timepoints: −24, −21, −18 (blank samples), 0.25, 0.5, 0.75, 1, 1.5, 2, 3, 4, 6, 8, 12, 14, 16, 24, 36, 48, 72, 96, 120, 144 and 168 h after treatment. Plasma was separated after centrifugation (10 min at 1400 × g) immediately after withdrawal. Three blank urine samples (sampled during spontaneous emiction) were taken from each horse between 24 and 18 h before treatment. Urine samples were taken at 2, 5, 7, 12, 24, 36, 48, 72, 96, 120, 144, 168 and 192 h after treatment for each dosage tested; for 50 mg/kg ASA, an additional sample was taken after 216 h. Both, urine and plasma samples were stored at −20 °C until analysis (storage time about 4 weeks).

#### Quantification of SA in urine and plasma

Initially, it had been planned to measure ASA and SA in urine and plasma samples. However, this this was not feasible as ASA turned out to be sensitive to methanol, heat, change of pH and was continuously dissociated to SA, even during LC-MS analysis. ASA could therefore not be detected with sufficient accuracy so that it was decided to convert all ASA to SA and to measure total salicylates in plasma and urine by increasing the pH to 13–14. Since SA is the main metabolite of ASA, no other metabolites such as gentisic or salicyluric acid were quantified. Quantification of SA was partially based on methods described previously [11] and accomplished by an internal standard calibration. SA concentrations were determined using chromatographic peak area/concentration ratios and linear regression analysis to IS area ratios.

#### Materials and chemicals

Ammonium acetate, glacial acetic acid, potassium hydroxide, sodium dihydrogen phosphate-monohydrate, di-sodium hydrogen phosphate and methanol (analytical grade) were obtained from Merck (Darmstadt, Germany); acetonitrile (HPLC grade) was purchased from VWR (Darmstadt, Germany). Oasis ® HLB SPE cartridges (60 mg, 3 mL) were purchased from Roche (Mannheim, Germany). Deionised water was of MilliQ grade. SA and the internal standard D_4_-SA were obtained from Sigma-Aldrich (Germany) and Toronto Research Chemicals (North York, Canada), respectively. For standard curves, pooled urine of horses with known SA concentrations as well as commercially available equine donor plasma (Sera Laboratories International, West Sussex, UK) were used.

#### Plasma sample preparation

For plasma samples, a direct injection method published by Thomas et al. [12] was modified. To 500 μL Milli-Q-water and 1 μg of the internal standard D4-SA 500 μl plasma were added. Samples taken up to 6 h (12.5 and 25 mg/kg) and up to 8 h after ASA administration were diluted 1:5 in Milli-Q-water before sample preparation. For protein precipitation, 1.5 mL acetonitrile were added and gently mixed. After centrifugation (10 min, 3000 U), 20 μL of KOH (5 mol/L) were added to the supernatant to alkalinize the sample to pH 13–14 for 20 min in order to hydrolyze all ASA to SA. To make the pH compatible with the HPLC column, the sample was adjusted to pH 1–2 by adding 20 μL HCl (6 mol/L) and centrifuged again (10 min, 1400 g). 200 μL aliquots were used for HPLC-MS/MS analysis.

#### Urine sample preparation

The sample preparation for the quantitative analysis of SA was performed following the method described by Schenk et al. [11] and included a solid phase extraction. Briefly, 2 μg of the internal standard D4-SA were added to 100 μL of urine and 900 μL of Milli-Q-water. Samples taken during the first 24 h after treatment were diluted 1:10 in Milli-Q-water (12.5 mg/kg and 25 mg/kg), whereas samples of the 50 mg/kg group were diluted 1:50. To enforce hydrolysis of any remaining ASA to SA, the pH was adjusted to 13–14 by addition of 40 μL KOH (1 mol/l). After 20 min an adjustment to pH 7 was achieved by addition of 0.2 mL phosphate buffer (Na_2_HPO_4_/NaH_2_PO_4_,0.8 mol/l). After centrifugation (5 min, 500 g), solid phase extraction was performed with conditioned Oasis® HLB 3 cc (60 mg) extraction cartridges (Waters corp., Milford, MA, USA). Samples were then evaporated to dryness in a rotary evaporator and dried residues dissolved in 200 μL ammonium acetate/acetonitrile (30:20, v/v) for HPLC-MS/MS injection.

#### Instrumentation-liquid chromatography

The liquid chromatography system comprised an Agilent Series 1100 LC (Agilent Technologies, Waldbronn, Germany). Analyte separation (plasma and urine samples) was achieved with a Nucleodur Pyramid column (70 × 4 mm, 5 μm particle size) from Macherey-Nagel (Düren, Germany). For plasma samples, a Gemini C_6_ Phenyl (4 × 2 mm) guard column was added (Phenomenex, Aschaffenburg, Germany). The mobile phase comprised ammonium acetate buffer (5 mmol/l ammonium acetate, 0.1% glacial acid in MilliQ water, pH 3.5; solvent A) and acetonitrile (solvent B). The following programmed mobile phase gradient was used for analyte separation: gradient B 0–100% in 7 min, held for 1 min at 100% B, reequilibration time at 0% B for 3 min, run time 11 min. The mobile phase flow rate was 800 μL/min. The retention time was 5.2 min.

#### Instrumentation-mass spectrometry

Mass analysis was performed on an API 3200 triple-quadrupole mass spectrometer (AB Sciex, Darmstadt, Germany), equipped with an electrospray ionisation (ESI) interface. Samples were measured in the negative operation mode at an interface temperature 450 °C with an ion spray voltage of −4500 V. Collision-induced dissociation with nitrogen was performed at a collision gas pressure of 2.9 × 10^−3^ Pa. Diagnostic ions were detected in the multiple reaction monitoring mode (MRM). The transition ions monitored for SA were m/z 137 → −93; m/z 137 → −65; m/z 137 → −41; m/z 137 → −75; those for d_4_-SA were m/z 141 → −97; and m/z 141 → −69. The quantifying ion for urine samples were m/z 137 → −75 (collision energy −38 eV) and m/z 137 → 65 (collision energy −40 eV) for plasma, respectively. Data acquisition and analysis were accomplished with Analyst® software (version 1.4.2, AB Sciex).

#### Method validation

The method was validated according to the guidelines of the European Horseracing Scientific Liaison Committee [13]. Validation parameters were selectivity, recovery, linearity, limit of quantification, limit of detection, analyte stability, precision, and accuracy. The calibration range was 5 to 250 μg/mL (urine samples) and 0.3 to 20 μg/mL (plasma samples).

Recovery was only calculated for urine, as plasma concentrations were determined by direct injection. To prove stability, quality control samples were stored under the same conditions as post administration samples for a minimum of 4 weeks.

#### Pharmacokinetic analysis

Pharmacokinetic parameters of SA in plasma were calculated with WinNonlin® 5.3 (Pharsight, Mountain View, USA), using a non-compartmental analysis. Because the SA concentration in plasma samples of untreated horses was below of the LLOQ (0.3 μg/ml), the absolute values were used for the PK calculation. The following information was obtained: C_max_, T_max_, clearance (Cl/F), MRT, elimination rate constant, half-life λ_z_ and AUC_last_.

### Pharmacodynamic study, COX-1 assay, COX-2 assay

#### Materials and chemicals

Compounds used for the pharmacodynamic study were ASA and SA (all Sigma Aldrich, Munich, Germany). Substances were diluted in dimethyl sulfoxide (DMSO; Merck, Darmstadt, Germany) in concentrations from 0.1 to 1000 mmol/L. LPS (*Escherichia coli* O111:B4) used for COX-2 assays was obtained from Sigma Aldrich, Munich, Germany. Samples were analyzed for thromboxane B_2_ and prostaglandin E_2_ concentrations using enzyme immunoassays (Cayman Chemicals, Ann Arbor, MI, USA).

#### Animals and study design

According to Brideau *et al*. [14] and McCann et al. [15], the COX-1 inhibition was quantified by each substance’s ability to inhibit the formation of clot-induced Thromboxane B_2_ (TXB_2_) using blood from six clinically healthy warmblood horses (five mares and one gelding). To assess COX-2 inhibition, LPS-induced Prostaglandin E_2_ (PGE_2_) production was measured.

#### In vitro assay

For the COX-1 assay, blood was drawn by jugular venipuncture into vacuum tubes containing no anticoagulant (Greiner bio-one, Frickenhausen, Germany). Immediately afterwards, blood aliquots (500 μL) were transferred into polypropylene tubes prepared with 5 μL of vehicle (DMSO), ASA or SA at final concentrations of 0.1, 1, 10, 100, or 1000 μmol/L. After mixing, tubes were incubated for 1 h at 37 °C to allow the blood to clot. Samples were then centrifuged at 4 °C and 2000 × g for 10 min. Supernatants were stored at −80 °C until analysis.

For the COX-2 assay, plasma was drawn in lithium heparin tubes (Vacutainer, BD, Heidelberg, Germany). Aliquots of 500 μL were transferred into polypropylene tubes and preincubated with 10 μL LPS dissolved in phosphate buffered saline (100 μg/mL). After 5 min of incubation at 37 °C, ASA or SA were added. A further incubation period of 24 h at 37 °C followed. One aliquot of blood was not incubated with LPS and used as control. Samples were centrifuged as described above and supernatants stored at −80 °C. A pre-incubation with a COX-1 inhibitor was not included in the performed COX-2 assay. After thawing, samples were diluted in EIA buffer (1:10) and used directly for the immunoassays without a preliminary extraction. The immunoassays were performed according to the manufacturer’s instructions (Dynatech Microplate Reader, Dynatech Laboratories, Denkendorf, Germany).

#### Statistical analysis

Data were analyzed with a commercially available software program (GraphPad Prism 5.03 software; GraphPad Software, Inc., La Jolla, CA, USA) by use of a one-way-repeated measures analysis of variance followed by the Bonferroni *post hoc* test. Values of *P* < 0.05 were considered statistically significant. The concentration leading to a 50% inhibition of COX activity (IC_50_) was calculated with WinNonlin® Professional Edition, Version 5.3, Inhibitory Effect Sigmoid Imax Model (Pharsight, Mountain View, USA).). The vehicle control was used as baseline (0% inhibition).

## Results

### Validation of the analytical method

Identification of SA was ensured by its specific retention time and four characteristic ion transitions. As no SA free horse urine and plasma was available, traces of SA could be detected in each sample. Nevertheless, the SA concentrations were mostly below the LLOQ and could easily be discriminated from the spiked samples. Plasma and urine samples spiked with SA that had been stored under the same conditions as the post administration samples, storage at −20 °C for four weeks did not show any significant difference in analyte degeneration (one-tailed *T*-test). Recovery was calculated to be 51% in urine.

Calibration curves were found linear in plasma and urine relating to the specified concentration ranges. The LLOD was estimated at 1 μg/mL for urine and 0.1 μg/mL for plasma. The LLOQ was determined at 5 μg/mL for urine and 0.3 μg/mL for plasma. Summary results for precision and accuracy are listed in Table 1.

**Table 1:** Precision and accuracy of the analytical method, summary results for plasma and urine

Concentration (μg/ml)	Intraday precision (%) (*n* = 6 per conc.)	Interday precision (%) (*n* = 18 per conc.)	Accuracy (%) (*n* = 6 per conc.)
Plasma			
1	4.6	10.3	2.3
5	4.8	1.1	4.8
10	3.1	3.4	1.6
Urine			
10	5.1	13.0	6.3
50	3.4	4.5	5.1
200	8.8	3.2	2.2

### Plasma and urine concentrations of SA after oral ASA administration

12.5 mg/kg ASA: Maximum plasma concentrations (C_max_)between 14.5 and 26.9 μg/mL were measured 0.5 h to 1.5 h after administration of ASA. Only in one horse C_max_ was reached eight hours after treatment. Plasma concentrations fell below the set threshold of 6.5 μg/mL between 6 and 16 h after treatment. Basal SA levels were measured 36 to 48 h after treatment (Fig. 1). In urine, maximum SA concentrations were achieved between 2 and 7 h after administration of ASA, with results varying between 699 and 10200 μg/mL. Values fell below the threshold of 750 μg/mL between 7 and 26 h after administration. One horse did not exceed the urine threshold SA at all (Fig. 2).

**Fig. 1:** Mean values (± S.D.) of SA concentrations in plasma of horses after a single oral dose of 12.5 mg/kg BW (*n* = 8). Black line = values > LLOQ. Grey line = values < LLOQ. Dotted line = LLOQ. Dashed line = threshold concentration (FEI)

**Fig. 2:** Mean values (± S.D.) of SA concentrations in urine of horses after a single oral dose of 12.5 mg/kg BW (*n* = 8). Black line = values > LLOQ. Grey line = values < LLOQ. Dotted line = LLOQ. Dashed line = threshold concentration (FEI)

25 mg/kg ASA: C_max_ was reached between 0.5 and 6 h after administrartion (19.1 to 37.8 μg/mL), while plasma concentrations dropped below the threshold of 6.5 μg/mL SA between 12 and 24 h. Between 36 and 48 h after treatment basal levels were reached in all horses (Fig. 3). All horses showed the highest urinary excretion of SA between 2 and 5 h after treatment, with values from 1550 to 7640 μg/mL SA. Between 7 and 24 h after administration, all horses featured urine SA levels below the threshold (Fig. 4).

**Fig. 3:** Mean values (± S.D.) of SA concentrations in plasma of horses after a single oral Black line = values > LLOQ. Grey line = values < LLOQ. Dotted line = LLOQ. Dashed line = threshold concentration (FEI)dose of 25.0 mg/kg BW (*n* = 8)

**Fig. 4:** Mean values (± S.D.) of SA concentrations in urine of horses after a single oral dose of 25.0 mg/kg BW (*n* = 8). Black line = values > LLOQ. Grey line = values < LLOQ. Dotted line = LLOQ. Dashed line = threshold concentration (FEI)

50 mg/kg ASA: Plasma SA levels peaked between 1 and 6 h after administration (35.1 to 62.7 μg/mL). Plasma levels fell below the threshold at 12 h (*n* = 2), 14 h (*n* = 1), 24 h (*n* = 3) and 36 h (*n* = 2) after administration. Basal levels could be observed again between 36 and 48 h after administration (Fig. 5). Peak urine SA concentrations were measured between 2 and 7 h (2810 to 9640 μg/mL). Values fell below the threshold between 12 and 36 h (Fig. 6).

**Fig. 5:** Mean values (± S.D.) of SA concentrations in plasma of horses after a single oral dose of 50.0 mg/kg BW (*n* = 8). Black line = values > LLOQ. Grey line = values < LLOQ. Dotted line = LLOQ. Dashed line = threshold concentration (FEI)

**Fig. 6:** Mean values (± S.D.) of SA concentrations in urine of horses after a single oral dose of 50.0 mg/kg BW (*n* = 8). Black line = values > LLOQ. Grey line = values < LLOQ. Dotted line = LLOQ. Dashed line = threshold concentration (FEI)

A plasma clearance (Cl/F) of 82.2 mL∙h/kg, resulting in a calculated half-life of 5.2 h (12.5 mg/kg), 97.1 mL∙h/kg with a half-life of 5.0 h (25 mg/kg), and 114.0 mL∙h/kg with a half-life of 5.7 h (50 mg/kg) were calculated (Table 2). The MRT varied between 7.26 and 8.39 h.

**Table 2:** Plasma SA pharmacokinetics data after oral administration of ASA (12.5, 25.0, 50.0 mg/kg) to horses, mean ± S.D. of eight horses per treatment

Parameter	Units	12.5 mg/kg	25.0 mg/kg	50.0 mg/kg
Cmax	μg/ml	19.75 ± 5.22	30.06 ± 7.44	51.66 ± 11.27
Tmax	h	2.0 ± 2.5	2.5 ± 2.3	2.2 ± 1.7
CI/F	ml/h/kg	82.2 ± 18.4	97.1 ± 19.9	114.0 ± 31.9
AUC*last*	h x μg/ml	154.9 ± 31.8	264.9 ± 63.2	457.1 ± 114.8
λZ	1/h	0.145 ± 0.040	0.148 ± 0.041	0.145 ± 0.061
λZ T½	h	5.1 ± 1.4	5.0 ± 1.3	5.7 ± 2.8
MRT	h	7.26 ± 2.13	7.81 ± 1.70	8.39 ± 3.67

### Pharmacodynamic study

In order to determine IC_50_ values, the inhibition of COX-1 and COX-2 activity was plotted against different concentrations of ASA (Table 3 and Fig. 7). The vehicle control was used as the baseline (0% inhibition). The IC_50_ of ASA was 1.68 μmol/L (0.50 μg/mL, COX-1) and 17.02 μmol/L (5.14 μg/mL, COX-2), respectively. No IC_50_ could be calculated for SA because of an insufficient COX-Inhibition (IC_50_ > 100 μmol/L (COX-1) and > 1000 μmol/L (Cox-2)).

**Table 3:** Inhibition of COX-1 and COX-2 activity (%) by ASA and SA; calculated based on in vitro assays (mean ± S.D. of experiments with equine blood samples of 6 horses)

Concentration (μmol/l)	ASA		SA	
	COX I	COX II	COX I	COX II
0.1	9.1 ± 3.6	9.8 ± 4.6	19.6 ± 9.5	4.7 ± 2.3
1.0	30.8 ± 16.0	12.6 ± 8.3	13.0 ± 5.7	15.3 ± 9.3
10.0	87.0 ± 11.5	37.9 ± 29.3	22.8 ± 10.0	10.3 ± 3.4
100.0	93.6 ± 10.3	60.9 ± 23.4	32.2 ± 21.1	–4.7 ± 3.2
1000.0	92.7 ± 12.9	75.7 ± 32.7	65.8 ± 28.4	26.8 ± 11.3

**Fig. 7:** Inhibition of COX-1 (black line) and COX-2 (dashed line) by ASA as a result of in vitro assays performed with equine blood; mean ± S.D. of 6 single experiments

## Discussion

A method for the quantitative analysis of SA in horse urine and plasma has been developed and validated. Because of the distinctive instability of ASA during the whole process of sample storage, preparation and analysis, it was decided to convert ASA completely to SA. Thus the origin of analysed SA values may be caused by a medication with SA or ASA which is metabolized to SA as well as by SA as a feeding component of plant origin (alfalfa hay, willow bark). With a LLOD (LLOQ) of 0.1 μg/mL (0.3 μg/mL) plasma the method is sensitive enough to detect an ASA administration, because mean population values of SA were reported to be about 0.23 μg/mL. The LLOD (LLOQ) for urine was determined to be 1 (5) μg/mL which is adequate considering the high mean population value of 27.3 μg/mL [11]. The SA concentration in plasma and urine samples (blanks) of the horses used in the described study was less than 0.3 μg/mL plasma and between <5 and 51 μg/mL urine.

According to our data, ASA inhibits COX-1 more potently than COX-2, with IC_50_ values of 1.68 μmol/L and 17.02 μmol/L, respectively. This finding is supported by the fact that ASA is known to only inhibit COX-1 irreversibly [16, 17]. The IC_50_ values calculated for ASA confirm results from other non-equine where ASA IC_50_ values from 1.67 to 4.45 μmol/L for COX-1 and from 5.34 to 15.9 μmol/L for COX-2 were described [18–21]. On the contrary, Vane and Botting [22] calculated an ASA IC_50_ of 278 μmol/L for COX-2. SA did not inhibit either COX effectively enough to calculate an IC_50_ value for the concentrations used in this study (up to 1000 μmol/L). Similar findings have been reported in other studies [18, 19, 21]. However, since SA does have a clinically proven effect [23] there has to be another mode of action. An action trough NF-κB or gentisic acid is just mentioned, but no specific role of these factors has been proposed to explain the anti-inflammatory activity of SA [21, 24].

In doping control the international threshold for SA in plasma is 6.5 μg/mL. This means that a SA confirmation may only be reported as “positive” if the detected concentration is above this limit. A SA concentration above this threshold can not be explained by SA as a feeding component. Measuring SA concentrations below the threshold level, it remains unclear if the measured SA concentration is caused by an ASA or SA medication or by SA as a feeding component [5, 11]. The presented excretion study should give evidence in how far this threshold is exceeded after a therapeutic medication of ASA.

The threshold was exceeded by 30 min and eight 8 h following oral administration of 25 and 50 mg/kg ASA, respectively. Twenty-four hours after administration of 25 mg/kg and thirty-six hours after administration of 50 mg/kg plasma concentrations of all horses were below the threshold again. The lower dosage of 12.5 mg/kg which may be used because of the antithrombotic effects of ASA, led to “positive” concentrations for 12 h after administration. Thus the detection period of an ASA administration in a blood sample is rather short.

The detection of an ASA medication is even more difficult in urine samples when applying the urine threshold of 750 μg/mL. Concentrations higher than this level were only detected for 24 h after the 50 mg/kg and for 12 h after administration of the 25 or 12.5 mg/kg dose. After administration of 12.5 mg/kg one horse did not exceed the threshold at all.

As the detection period of an ASA medication (time of SA above the threshold) is less than one day in almost all horses of our study, it has to be discussed whether its therapeutic effect can be controlled adequately with the existing rules.

Broome et al. [4] described a rapid decline of the ASA concentration after intravenous administration of 20 mg/kg ASA to horses. The ASA concentration was below 0.1 μg/mL after four hours [4]. Comparing the ASA concentrations measured by Broome et al. (2003) with the IC_50_ values calculated in the described study, it can be concluded that a COX-1 inhibitory effect may be reached for a period of about 3 to 4 h. A COX-2 inhibition should be expected for only 1.5 h. There are hints that salicylates accumulate in synovial fluid after systemic administration, as demonstrated *in vitro* by Friebe et al. [25] who simulated a systemic ASA treatment with 20 mg/kg I.V. in the isolated perfused equine distal limb. Extrapolated from synovial fluid concentrations measured in *vitro*, a COX-1 inhibitory effect can be expected in the joint for about 6 to 8 h (COX-1) and 2 h (COX-2). The results of the *in vitro* and *in vivo* studies [26] indicate that even if SA values in plasma and urine fall below the thresholds, one cannot exclude any therapeutic effect, especially since NSAIDs are generally known to accumulate in inflammatory exudate [27].

## Conclusion

The established SA thresholds of 750 μg//mL urine and 6.5 μg/mL plasma appear too generous and are leaving space for misuse of the anti-inflammatory and analgetic compound ASA especially for countries where horse feed is not naturally rich in salicylates.

## Abbreviations

ASA: Acetylsalicylic acid
COX: Cyclooxygenase
DMSO: Dimethyl sulfoxide
FEI: International Equestrian Federation
HPLC-MS/MS: High performance liquid chromatography–mass spectrometry
LLOQ: Lower limit of quantification
LPS: Lipopolysaccharide
PGE: Prostaglandin E
SA: Salicylic acid
TXB: Thromboxane B
